# Effectiveness of Multidisciplinary Nursing Based on Fever, Blood Sugar, and Swallowing Function Management in Patients with Acute Stroke

**DOI:** 10.1155/2022/5949760

**Published:** 2022-06-21

**Authors:** Dannan Ai, Yifang Gu, Sumin Xu

**Affiliations:** ^1^Emergency Department, The First Affiliated Hospital of Soochow University, Suzhou, China; ^2^Interventional Department, The First Affiliated Hospital of Soochow University, Suzhou, China

## Abstract

**Purpose:**

The aim of this study was to assess the effectiveness of multidisciplinary nursing based on fever, blood sugar, and swallowing function management in patients with acute stroke (AS).

**Methods:**

A total of 200 AS patients who were treated in our hospital from January 2016 to January 2020 were recruited and randomized at a ratio of 1 : 1 into a control group and a study group. The control group received standardized early rehabilitation nursing, and the study group received multidisciplinary nursing based on fever, blood sugar, and swallowing function management plus standardized early rehabilitation nursing. The patients were also assigned different blood glucose levels upon admission to a high blood glucose group or a normal blood glucose group. The clinical endpoint is clinical efficacy.

**Results:**

Multidisciplinary nursing resulted in better clinical outcomes and treatment efficiency in the patients in the study group versus standardized early rehabilitation nursing. When compared with the control group, the patients in the study group showed lower National Institute of Health Stroke Scale (NIHSS) scores, higher Barthel Index (BI) scores, lower fasting blood glucose levels and body temperature 24 hours after admission, a lower incidence of swallowing dysfunction and aspiration pneumonia 30 days after nursing, and lower C-reactive Protein (CRP) levels 7 days after nursing. The NIHSS scores of the high blood glucose group were significantly higher than those of the normal blood glucose group.

**Conclusion:**

Multidisciplinary nursing based on fever, blood sugar, and swallowing function management for patients with AS improves the clinical outcome and treatment efficiency, restores the swallowing function and blood glucose level, and ameliorates the long-term prognosis of patients.

## 1. Introduction

Acute stroke (AS) is an acute cerebrovascular disease and is caused by the sudden rupture of blood vessels in the brain or the insufficiency of blood flow into the brain due to vascular obstruction, with high morbidity, disability, and mortality [1, 2]. The goal of the AS treatment is to minimize functional disorders, restore limb function and cognitive ability, prevent complications, and enhance the patients' prognosis [3, 4]. Therefore, effective nursing regimens are of great significance to lower the disability rate and improve the quality of life of patients. Early rehabilitation nursing with a stroke unit as the main model has been widely used in stroke nursing. A previous study has suggested that traditional Chinese medicine (TCM) physiotherapy for dysphagia patients after stroke could improve the swallowing-related muscle function and muscle amplitude and shorten the swallowing time [5]. The onset of AS is associated with a strong stress response, which causes aberrant changes in body temperature and blood sugar, and delayed treatment may result in a compromised prognosis for patients [6]. In addition, swallowing dysfunction is a common sequela of stroke and may lead to serious complications such as aspiration pneumonia [7]. The present study was conducted to assess the effectiveness of multidisciplinary nursing based on fever, blood sugar, and swallowing function management in patients with AS.

## 2. Materials and Methods

### 2.1. General Information

A total of 200 AS patients who were treated in our hospital from January 2016 to January 2020 were recruited and randomized into a control group and a study group, with 100 cases in each group.

### 2.2. Inclusion and Exclusion Criteria

Inclusion criteria: patients who were diagnosed with AS by clinical and imaging examinations [8]; aged 18–80 years; with a time-lapse from onset to randomization within 6–12 h; with tolerance to nursing measures such as oral examination and sampling; and who provided written informed consent after being fully informed of the purpose and process of the study were included.

Exclusion criteria: patients with a history of brain tumors, encephalitis, epilepsy, and demyelinating diseases of the nervous system; with a history of traumatic brain injury in the past 3 months; who were pregnant or lactating; with severe heart, lung, liver, kidney, blood system, and other diseases; and with mental disorders or a history of dementia were excluded. This study was approved by the ethics committee of the First Affiliated Hospital of Soochow University, with an approval number of 2016SD (113).

### 2.3. Nursing Methods

The control group received standardized early rehabilitation nursing. (1) *Position Placement and Passive Movement*. The patients were instructed and assisted to maintain the correct posture and position of the limbs to prevent limb contractures and joint deformations, given their unstable vital signs in the early stage. After the vital signs were stabilized, the passive joint movement exercise was performed to maintain muscle tension and joint mobility if the patients failed to achieve active mobility. Movements of flexion, extension, adduction, abduction, and rotation were performed in the normal range of joint activities, with a sequence of passive movements from large joints to small joints and a range of motion from small to large. Violent stretching and strenuous exercise were avoided, and massage and relevant methods were also performed to promote local blood circulation, eliminate pain, and prevent complications such as bedsores, shoulder-hand syndrome, and phlebitis. (2) *Early Activities and Physical Therapy*. The motor relearning program was used and the patients were encouraged to receive early rehabilitation training. On the theoretical basis of the functional reorganization of the central nervous system in neurophysiology, a scientific motor relearning program was used to boost the recovery of motor function. Specifically, the motor relearning program includes 7 items, namely, upper limb function training, oral and facial function training, sitting up to the bedside training, sitting balance training, standing sitting training, standing balance training, and walking training. Furthermore, balance and gait posture training and strength training were also carried out. Early rehabilitation training should follow the principle of individualization, step by step, once a day, no more than 40 minutes each time. (3) *Psychological Rehabilitation Nursing*. The environment of the ward was kept quiet, tidy, and warm. The symptoms of patients such as sensory impairment, slowness of movement, and language impairment were closely monitored, and the patients were encouraged to communicate with others to eliminate negative emotions.

The study group received multidisciplinary nursing care based on fever, blood sugar, and swallowing function plus standardized early rehabilitation nursing. (1) *Body Temperature Care*. A multidisciplinary collaborative team was established, including internists, convalescents, psychological consultants, and TCM physiotherapists, which is jointly responsible for the assessment of the patient's condition, swallowing function, and psychological status; the development of nursing programs; and the delivery of professional training and guidance. Within 72 hours after admission, the patients' body temperatures were monitored and recorded hourly. Paracetamol was applied if the temperature exceeded 37.5°C. (2) *Blood Sugar Management*. On admission, venous blood glucose was measured. Within 72 hours after admission, the fingertip blood glucose assay was performed hourly, and diabetic patients with a blood glucose level of 8–11 mmol/L or nondiabetic patients with a blood glucose level of 8–16 mmol/were given an intravenous infusion of normal saline for 6 hours. Within 48 hours of admission, diabetic patients with blood glucose greater than 11 mmol/L or nondiabetic patients with blood glucose greater than 16 mmol/received intravenous insulin to control their blood glucose level below 8.3 mmol/L. (3) *Swallowing Function Nursing*. All patients received swallowing dysfunction screening, the nurses received swallowing function nursing training, and the swallowing function training was performed on patients, including ice stimulation and empty swallowing, glottis closing training, and swallowing-related muscle training. (a) Ice stimulation and empty swallowing: the nursing staff used the tip of a frozen brush to dip a little ice water and apply it gently to the patients' anterior and posterior palatal arch, soft palatal arch, posterior pharyngeal wall, and the back of the tongue for stimulation, so as to sensitize the areas that trigger the swallowing reflex and strengthen the swallowing reflex. The stimulation was immediately stopped in the presence of a vomiting reflex to avoid choking and aspiration. (b) Glottis closing training: the training of cough and breath-holding vocal movement was performed to prevent and reduce the entry of food into the trachea. (c) Swallowing-related muscle training: it included the training of the tongue muscle, soft palate elevation, and laryngeal muscle training. When aspiration was detected, the patient was placed in a prone position immediately, with the head low and the feet high, and the nursing staff tapped the back of the patient to discharge the phlegm. Acupressure was performed on the acupuncture points of Xiaguan, Jiache, Dayin, Dicang, Lianquan, Chenggrong, Fengchi, Quchi, and Hegu.

### 2.4. Observational Indicators

#### 2.4.1. Clinical Outcome

The modified Rankin scale [9] (mRS) was used to evaluate the 30-day clinical outcome. The mRS is divided into 0–6 points, with completely asymptomatic for 0 points, symptomatic but no obvious dysfunction for 1 point, mildly disabled with complete self-care ability for 2 points, moderately disabled with partial self-care ability and no need of assistance during walking for 3 points, severely disabled and unable to walk independently for 4 points, severely disabled and bed rest for 5 points, and death for 6 points. A mRS score of ≤2 points was considered a positive outcome, and a score of ≥3 points was considered a poor outcome.

#### 2.4.2. Neurological Function and Quality of Life Score

The NIHSS score [10] was used to evaluate neurological function and clinical efficacy. The NIHSS contains assessments of consciousness, language, movement, sensation, mutual aid movement, eye movement, and visual field, with a score of 0–42 points. The higher the score, the more severe the neurological deficit. According to the NHISS score and mRS score, the clinical efficacy was divided into four levels: basically cured, significantly improved, partially improved, and ineffective. The efficacy was considered cured if the NIHSS score was reduced by ≥90%. The efficacy was considered significantly improved if the NIHSS score reduction was between 45% and 90%. The efficacy was considered partially improved if the NIHSS score reduction was between 18% and 45%, and the efficacy was considered ineffective if the NIHSS score was reduced by ≤8%. Efficiency = (cured + significantly improved + partially improved)/total number of cases × 100%. The Barthel Index (BI) was used to assess the quality of life of patients. The BI score includes 10 items, including 8 items of self-care activities (eating, grooming, toileting, bathing, dressing and undressing, walking, and urine control) and 2 items of mobility-related activities (walking 50 m on flat ground or in a wheelchair, and walking up and down stairs). The BI score totals 100 points. The higher the score, the stronger the autonomy of life and the lower the dependence.

#### 2.4.3. Swallowing Function

The swallowing function of patients was divided into 5 grades using the Kubota Drinking Water Test [11]. The patients took a sitting position or a 30° lying position and drank 30 mL of warm water. Grade I: the patient drank up the water once within 5s without choking; Grade II: the patient finished drinking the water twice or more without choking; Grade III: the patient drank up the water once with choking; Grade IV: the patient finished drinking the water twice or more with choking; and Grade V: the patient failed to drink up the water with obvious choking. Grades I and II refer to full swallowing function, and Grades III to V refer to swallowing dysfunction.

#### 2.4.4. Blood Glucose Level and Temperature Control

The fasting blood glucose of the two groups of patients was determined on the day after admission and 3 days after nursing, and their body temperature was monitored. Fasting blood glucose of over 11.1 mmol/L was defined as high blood glucose.

#### 2.4.5. Aspiration Pneumonia and C-Reactive Protein

During the nursing, the patients' status and the proportion of patients with aspiration pneumonia within 30 days were monitored. Diagnostic criteria for aspiration pneumonia: no previous history of bronchial diseases or lung diseases; coughing, shortness of breath, cyanosis, sputum, fever for more than 3 days after stroke; dry and wet rales in both lungs; and body temperature >37°C. Blood routine indexes: white blood cells >11 × 109/L and neutrophil ratio >0.70; scattered irregular patchy opacity in both lungs with blurred edges by lung CT or *X*-ray chest radiographs. In addition, 30 days after nursing, fasting venous blood was collected from the patients, and the serum C-reactive protein (CRP) concentration of the patients was determined by an enzyme-linked immunosorbent assay (ELISA), with CRP ≤ 5 mg/L as the normal value.

### 2.5. Statistical Methods

In this research, SPSS23.0 was used for data analysis, and GraphPad Prism 8.0 (GraphPad Software, San Diego, USA) was used to plot the graphics. The measurement data are represented by (mean ± SD), and the count data are represented by (*n* (%)). A two-sample independent *t*-test was used for comparison of measurement data, a paired *t*-test was used for comparison at different time points within the group, and chi-square analysis was used for count data comparison. *P* < 0.05 indicated that the difference was statistically significant.

## 3. Results

### 3.1. Comparison of General Data and Clinical Outcomes

As shown in Table 1, the two groups demonstrated no obvious disparity in general information (all *P* > 0.05). As shown in Figure 1, in the control group, there were 24 cases of 0 points, 26 cases of 1 point, 21 cases of 2 points, 13 cases of 3 points, 7 cases of 4 points, 7 cases of 5 points, and 2 cases of 6 points in terms of mRS scores, with 29 cases having a poor outcome. In the study group, there were 25 cases of 0 points, 33 cases of 1 point, 25 cases of 2 points, 8 cases of 3 points, 5 cases of 4 points, 3 cases of 5 points, and 1 case of 6 points in terms of mRS scores, with 17 cases having a poor outcome. The study group had better clinical outcomes than the control group (*P* < 0.05).

### 3.2. Comparison of Clinical Efficacy

In the control group, 26 cases were cured, 24 cases were significantly improved, 37 cases were partially improved, and 13 cases were ineffective, with a total clinical efficiency of 87%; In the study group, 37 cases were cured, 33 cases were significantly improved, 27 cases were partially improved, and 3 cases were ineffective, with a total clinical efficiency of 97%. The clinical efficacy was superior in the study group versus the control group (*P* < 0.05). (Table 2).

### 3.3. Comparison of NIHSS Score and BI Score

There were no significant differences between the two groups in terms of NIHSS score (16.84 ± 3.36 vs. 17.11 ± 2.04) (*P* > 0.05). 30 days after nursing, the study group showed a lower NIHSS score (7.93 ± 1.36) than the control group (10.76 ± 1.07) (*P* < 0.05). The two groups showed no significant differences in BI scores (31.08 ± 8.27 vs. 33.25 ± 7.79) (*P* > 0.05). 30 days after nursing, the study group had a significantly higher BI score (72.94 ± 14.82) than the control group (64.28 ± 12.47) (*P* < 0.05) (Figure 2).

### 3.4. Comparison of Blood Glucose Levels and Body Temperature

Before nursing, the two groups showed similar fasting blood glucose levels and body temperature (*P* > 0.05). 24 hours after nursing, patients in the control group showed significantly higher fasting blood glucose than those in the study group (*P* < 0.05). 72 hours after nursing, the blood glucose of the two groups showed a drastic decline (*P* < 0.05), and no intergroup difference was found (*P* > 0.05). At 24 hours and 72 hours after nursing, patients in the study group showed a lower body temperature than the control group (*P* < 0.05) (Tables 3 and 4).

### 3.5. Comparison of Swallowing Function and Incidence of Aspiration Pneumonia

As demonstrated in Table 5, in the control group, there were 34 cases of Grade I, 30 cases of Grade II, 17 cases of Grade III, 12 cases of Grade IV, and 7 cases of Grade V, with an incidence of swallowing dysfunction of 36%. In the study group, there were 45 cases of Grade I, 46 cases of Grade II, 5 cases of Grade III, 3 cases of Grade IV, and 1 case of Grade V, with an incidence of swallowing dysfunction of 9%. The incidence of swallowing dysfunction in the study group was significantly lower than that of the control group (*P* < 0.05). A total of 13 cases of aspiration pneumonia were recorded in all patients, and their swallowing functions were all categorized into Grades III to V, among which 1 case was Grade III, 3 cases were Grade IV, and 7 cases were Grade V. A lower incidence of aspiration pneumonia (2 cases) in the study group than that (11 cases) in the control group was observed (*P* < 0.05).

### 3.6. Comparison of CRP Levels

The two groups showed similar serum CRP levels before nursing (*P* > 0.05), and the serum CRP levels of both groups significantly declined at 15 days and 30 days after nursing, with lower results in the study group (*P* < 0.05). (Figure 3).

### 3.7. The Relationship between Different Blood Glucose Levels at Admission and the NIHSS Scores

As shown in Table 6, according to the results of venous blood glucose testing after admission, all patients were divided into the high blood glucose group (59 cases) and the normal blood glucose group (141 cases). The NIHSS score of the high blood glucose group was 13.68 ± 3.54, which was higher than that of 9.18 ± 3.82 in the normal blood glucose group (*P* < 0.05).

## 4. Discussion

Stroke is a major disabling disease for the elderly in China that seriously compromises the quality of life of patients and imposes a heavy economic burden on their families. Early rehabilitation therapy plays a key role in the functional recovery of stroke patients. Stroke causes a significant increase in body temperature, aggravates nerve damage, increases the area of infarction, and shortens the treatment window. Research has shown that for every 1°C increase in body temperature, the relative risk of adverse outcomes rises by 3.9 times [12]. Stress hyperglycemia is a protective response of the body to critical and severe diseases and injuries. Ineffective blood glucose control may aggravate the damage of the original disease, impair the immune function of the body, and cause infections, acid-base balance disorders, and organ failure [13]. Swallowing dysfunction is a common complication of stroke that is associated with eating difficulties, insufficient nutrient intake, aspiration pneumonia, and even death from suffocation [14]. In addition, dysphagia may aggravate the patients' negative emotions and lead to the collapse of patients' confidence, which hampers the nursing efficacy. Accordingly, early treatment of fever, blood sugar management, and swallowing function is essential to improve nursing efficacy.

In the present study, the study group received multidisciplinary nursing based on fever, blood sugar, and swallowing function management and achieved promising results, and the results showed that the clinical outcome and total effective rate of treatment in the study group were significantly better than those in the control group. The mRS score and BI score are used as indicators of the level of functional disability [15]. The NIHSS score accurately reflects the level of neurological deficits and is commonly used for efficacy evaluation of neurological treatments [16]. In the present study, the study group showed a higher proportion of patients with mRS score ≤2 points, lower NIHSS scores, and higher BI scores than the control group, indicating that multidisciplinary nursing has an excellent clinical effect and improves the clinical outcome of patients. Previous studies have demonstrated that the increase in body temperature of patients with AS after admission is an independent risk factor for the mortality of stroke. The higher the body temperature, the higher the mortality rate. Elevated body temperature is a common phenomenon after a stroke that leads to increased secretion of neurotransmitters such as glutamate, higher production of oxygen free radicals, and elevated secretion of lactic acid, resulting in damage to the blood-brain barrier and aggravated brain tissue damage. Nonetheless, the relationship between body temperature and stroke prognosis is still debated. It has been reported that a low body temperature within 6 hours after a stroke is associated with a poor prognosis [17]. Stroke causes a severe stress response in the body and promotes the secretion of glycogen hormones to enhance the resistance ability of the body, which results in changes in the internal environment and a stress-induced blood sugar increase [18]. In addition, iatrogenic supplementation of glucose solution and the use of glucocorticoids after hospitalization also trigger iatrogenic blood sugar elevation [19]. Hyperglycemia affects brain cell metabolism, aggravates the anaerobic glycolysis of infarcted tissues, promotes the release of excitatory glutamate, strengthens oxidative stress, and destroys the blood-brain barrier. This study confirmed that fever, blood sugar management, and swallowing function training could restore the body temperature, blood sugar, and swallowing function, thereby improving clinical efficacy.

## 5. Conclusion

The application of multidisciplinary comprehensive care based on fever, blood sugar, and swallowing function management for patients with AS improves the clinical outcome and treatment efficiency, restores the swallowing function and blood glucose level, and ameliorates the long-term prognosis of the patient, which is worthy of further promotion.

## Figures and Tables

**Figure 1:** Comparison of clinical outcomes.

**Figure 2:** Comparison of NIHSS scores and BI scores; ^*∗∗∗*^ indicates *P* < 0.001.

**Figure 3:** Comparison of CRP levels; ^*∗∗∗*^ indicates *P* < 0.001.

**Table 1:** Comparison of general information of the two groups of patients.

	Control group (*n* = 100)	Study group (*n* = 100)	*t*/*χ*^2^	*P*
*Gender*				
Male	68	56	3.056	0.080
Female	32	44		

Age (years)	68.56 ± 13.57	67.18 ± 11.84	0.766	0.444
<60	29	37	1.447	0.229
≥60	71	63		

*Types of AS*				
Ischemic stroke	23	29	0.936	0.333
Hemorrhagic stroke	77	71		
Onset time (h)	5.87 ± 1.35	5.59 ± 1.24	1.528	0.128
<6 h	69	77	1.624	0.203
>6 h	31	23		

**Table 2:** Comparison of clinical efficacy.

	Cured	Significantly improved	Partially improved	Ineffective	Total effective rate
Control group (*n* = 100)	26	24	37	13	87
Study group (*n* = 100)	37	33	27	3	97
*χ* ^2^					6.793
*P*					0.009

**Table 3:** Changes in blood glucose 72 hours after admission.

	After admission	24 hours after nursing	72 hours after nursing
Control group (*n* = 100)	10.24 ± 2.36	12.82 ± 3.47	7.98 ± 1.27
Study group (*n* = 100)	10.52 ± 2.83	10.82 ± 2.12	7.71 ± 1.09
*t*	0.760	4.918	1.613
*P*	0.448	<0.001	0.108

**Table 4:** Changes in body temperature 72 hours after admission.

	After admission	24 hours after nursing	72 hours after nursing
Control group (*n* = 100)	36.25 ± 0.75	36.87 ± 0.82	36.75 ± 0.73
Study group (*n* = 100)	36.42 ± 0.67	36.56 ± 0.71	36.52 ± 0.61
*χ* ^2^	1.690	5.858	2.418
*P*	0.093	0.005	0.017

**Table 5:** Comparison of swallowing function and incidence of aspiration pneumonia.

	I	II	III	IV	V	Incidence of dysphagia	Aspiration pneumonia
Control group (*n* = 100)	34	30	17	12	7	36	11
Study group (*n* = 100)	45	46	5	3	1	9	2
*χ* ^2^	21.35					20.09	6.664
*P*	<0.001					<0.001	0.009

**Table 6:** The relationship between different blood glucose levels at admission and the NIHSS scores.

	NIHSS scores	NIHSS grading		
		≤7 points	8∼20 points	>20 points
High blood glucose group (*n* = 59)	13.68 ± 3.54	16	29	14
Normal blood glucose group (*n* = 141)	9.18 ± 3.82	67	45	29
*t*/*χ*^2^	8.64	7.704		
*P*	<0.001	0.021		

## Data Availability

The datasets used during the present study are available from the corresponding author upon reasonable request.
